# The Link between *ANRIL* Gene RS4977574 Polymorphism and Common Atherosclerosis Cardiovascular Complications: A Hospital-Based Case-Control Study in Ukrainian Population

**DOI:** 10.1155/2022/8468202

**Published:** 2022-10-05

**Authors:** Polina V. Kniazkova, Viktoriia Yu. Harbuzova, Vladyslav V. Pokhmura

**Affiliations:** Department of Physiology and Pathophysiology with Medical Biology Course, Medical Institute of the Sumy State University, Sumy 40034, Ukraine

## Abstract

**Materials and Methods:**

195 patients with ACS, 200 patients with LAS, and 234 control subjects were enrolled in this case-control study. Real-time PCR was used for *ANRIL* rs4977574 genotyping. SPSS software package (version 17.0, IBM, USA) was used for data analysis.

**Results:**

A significant association between rs4977574 polymorphism and the risk of atherosclerosis and cardiovascular complications was found under the recessive model regardless of adjustment for nongenetic risk factors (OR = 1.551; *p* = 0.025). Moreover, the link between rs4977574 locus and serum levels of total cholesterol (*p* = 0.021) and LDL (*p* = 0.022) was detected. A separate analysis in subgroups demonstrated the association of rs4977574 polymorphism with increased risk of ACS under the recessive model (OR = 1.501; *p* = 0.048). No relation between rs4977574 site and LAS development was revealed (*p* > 0.05).

**Conclusion:**

Obtained data suggested that *ANRIL* rs4977574-GG genotype can be a possible genetic marker for the development of atherosclerosis and cardiovascular complications in Ukrainian population.

## 1. Introduction

Atherosclerotic lesion of the cardiovascular system is known to be the leading cause of death in the world. It is reported that 30 to 40% of all deaths in different countries are caused by cardiovascular complications of atherosclerosis [1, 2]. That is why today the efforts of many research centers are aimed at revealing the molecular genetic markers and detailed mechanisms of atherosclerosis development. Since 2007, a number of genome-wide association studies (GWAS) have been performed, which have shown a strong link between the human chromosome 9p21.3 region and the development of coronary artery disease (CAD) [3, 4], ischemic stroke [5], and peripheral arterial disease [6].

It is currently established that the three tumor suppressor genes (cyclin dependent kinase inhibitor CDKN2A/p16^INK4A^, CDKN2A/p14^ARF^, and CDKN2B/p15^INK4B^), the methyladenosine phosphorylase gene, and the gene of long noncoding RNA (lncRNA) ANRIL (antisense noncoding RNA in the INK4 locus) are localized both on the sense and antisense strands of the chromosome 9p21.3 region [7]. *ANRIL* is considered a key gene in this genomic locus in the context of atherosclerosis onset and development. Functional studies by Yari et al. showed a significant decrease in the expression of the ANRIL transcript EU741058 in the peripheral blood of CAD patients [8]. Cho et al. found a significant reduction in the formation of the ANRIL transcript DQ485454 in the endothelial cells of arteries affected by atherosclerosis [9]. Moreover, the positive correlation between atherosclerosis severity and expression of ANRIL transcripts EU741058 and NR_003529 in atherosclerotic plaques was revealed by Holdt et al. [10]. It has also been shown that the polymorphic loci of the 9p21.3 region with the highest contribution to the risk of CAD development are located exactly in the *ANRIL* gene [11].

The question of specific molecular mechanisms of lncRNA ANRIL is not yet fully disclosed. However, it is assumed that the main effects of ANRIL transcripts are carried out through the interaction with proteins of polycomb repressive complex 1 and 2 (PRC1 and PRC2). Ultimately, this leads to epigenetic *cis*-inactivation of the already mentioned tumor suppressor genes: p16^INK4A^, p14^ARF^, and p15^INK4B^ [12].

The *ANRIL* gene (official name: CDKN2B-AS1; Gene ID: 100048912) consists of 126307 nucleotide pairs (NC_000009.12) and contains at least 21 exons. To date, more than 25 different linear and circular ANRIL isoforms formed during transcription have been described [13]. As of September 2021, 50,580 polymorphic loci are located in the *ANRIL* gene (according to the NCBI: https://www.ncbi.nlm.nih.gov/snp/?term=CDKN2B-AS1). It is considered that the single nucleotide polymorphism (SNP) rs4977574 is one of the most significant in relation to the occurrence of cardiovascular diseases. The results of several GWASs have shown a strong link between this polymorphic site and CAD development [11, 14, 15]. A large number of case-control studies to investigate the association of the rs4977574 locus with the risk of CAD [16–18], myocardial infarction [19–21], ischemic stroke [20, 22], and hypertension [23] has also been performed. In addition, several meta-analyses have confirmed an association between the rs4977574 polymorphism and the risk of myocardial infarction and ischemic stroke [16, 22, 24–26].

Most of the mentioned studies have been performed in different populations of Asia and America. There is almost no information on the different allelic variants distribution of *ANRIL* rs4977574 polymorphism among Ukrainians. The question of the possible link between rs4977574 SNP and the risk of atherosclerosis complications in Ukrainian population is totally uncovered. That is why we decided to perform our study.

### 1.1. The aim

The aim of the present work was to test the possible association between *ANRIL* gene rs4977574 polymorphism and the development of acute coronary syndrome and large artery stroke in Ukrainian population.

## 2. Materials and Methods

### 2.1. Study Population

In sum, 629 unrelated Ukrainians were enrolled in this hospital-based study. All subjects were divided into case (395) and control (234) groups. The case group included 195 patients with acute coronary syndrome (ACS) and 200 patients with large artery stroke (LAS).

All ACS patients were treated in the cardiology department of the Sumy Regional Clinical Hospital for War Veterans and Sumy Regional Clinical Hospital. The diagnosis of acute myocardial infarction and unstable angina was established on the basis of clinical, ECG, and biochemical examination in accordance with the recommendations of the European Society of Cardiology [27]. LAS patients were registered at the dispensary in the outpatient department of the Sumy Clinical Hospital No. 5. The ischemic nature of the stroke was established according to the anamnesis, disease clinical picture, and results of the brain magnetic resonance imaging. The subtype of ischemic stroke was determined according to the TOAST criteria [28] on the basis of anamnesis, disease, clinical course, and results of ECG and ultrasound Doppler examination of the main head arteries.

Patients with cardiogenic shock, severe renal and hepatic failure, bronchial asthma, trauma or major surgery, acute or chronic inflammation in the acute stage, malignant tumors, and systemic diseases were excluded from the study. On the first day of hospitalization, serum lipid profiles (total cholesterol, HDL, LDL, and triglycerides) were determined in 195 ACS patients and 187 LAS patients. Thus, the analysis of the effect of rs4977574 polymorphism on lipid metabolism was performed in 382 patients.

The control group included relatively healthy patients who underwent routine checkup at the Sumy Clinical Hospital No. 5 and the Sumy Regional Clinical Hospital. The absence of cardiovascular pathology was confirmed by collecting anamnestic data, recording ECG, blood pressure, measuring, and studying of blood biochemical parameters.

The study was complied with the principles of the Helsinki Declaration and was approved by the Bioethics Commission of the Medical Institute of Sumy State University (number 1/11 12 November, 2018). All participants provided written informed consent before enrollment.

### 2.2. Genotyping

Blood leukocyte DNA was extracted using commercial GeneJET Whole Blood Genomic DNA Purification Mini Kit (Thermo Fisher Scientific, USA). The genotyping of *ANRIL* gene polymorphic site rs4977574 was performed by real-time polymerase chain reaction (Real-time PCR) using TaqMan assay C_1754681_10 (catalog number: 4351379). Allele A was determined using probe containing fluorescent dye VIC, allele G: fluorescent dye FAM. The volume of reaction system was 10 *μ*l, including 5 *μ*l Master Mix 2x, 3.25 *μ*l H_2_O, 0.25 *μ*l forward and reverse primers, and 1.5 *μ*l genomic DNA. The QuantStudio 5 Dx Real-Time instrument (Applied Biosystems, USA) was used for reaction. The amplification consisted of an initial 10 minute denaturation (95°C) followed by 45 cycles of amplification for 15 sec (95°C) and for 30 s (60°C).

### 2.3. Data Analysis

Mathematical data analysis was performed using the SPSS software package (Statistical Package for the Social Sciences, version 17.0, IBM, USA). Continuous data were checked for normality using the Kolmogorov-Smirnov test. All continuous variables are presented in the form of mean and standard deviation (M ± SD). The correspondence of the rs4977574 genotype frequency to the Hardy–Weinberg equilibrium was assessed using the Pearson *χ*^2^ test. Comparative analysis of the genotype distribution, as well as the distribution of other categorical variables between the tested groups, was also performed using the *χ*^2^-criterion. Student's *t*-test for two independent samples was used to compare the mean values between two groups. The mean values between the carriers of three different rs4977574 genotypes were compared using the ANOVA method with the subsequent Bonferroni post hoc test. To determine the risk of atherosclerosis complications depending on the specific rs4977574 genotype, the binary logistic regression was applied. Multivariable logistic regression was used to adjust the analysis for sex, age, body mass index, smoking habit, and hypertension. Values of *p* < 0.05 in all tests were considered as statistically significant.

## 3. Results

The general characteristics of the comparison groups are presented in Table 1.

It was shown that the mean age in the control group (66.1 ± 14.5) was significantly higher than in patients with atherosclerosis (61.4 ± 11.0; *p* < 0.001). This fact increases the reliability of control, as it reduces the likelihood of atherosclerosis complications in later periods of these individuals' lives. In return, the case group had significantly higher mean systolic blood pressure (*p* < 0.001), mean diastolic blood pressure (*p* < 0.001), mean fasting glucose (*p* < 0.001), the number of people with hypertension (*p* < 0.001), the number of people with overweight (*p* = 0.012), and smokers (*p* = 0.003). No difference in the ratio of subjects of different sexes between the two groups was found (*p* = 0.744).

The lipid profile parameters in patients with atherosclerosis complications are shown in Table 2.

The serum blood concentration of total cholesterol and LDL in patients with ACS was significantly higher than in LAS patients (*p* < 0.001). However, the difference in the level of HDL and triglycerides between ACS and LAS patients was absent (*p* = 0.113 and *p* = 0.890, respectively).

The distribution of *ANRIL* rs4977574 genotypes in the control group (G-allele frequency = 0.438), in the common case group (G-allele frequency = 0.516), in ACS patients (G-allele frequency = 0.528), and in LAS patients (G-allele frequency = 0.505) did not deviate from the Hardy-Weinberg equilibrium (*p* = 0.276, *p* = 0.052, *p* = 0.058, and *p* = 0.397, respectively).

Table 3 indicates the results of *ANRIL* gene rs4977574 genotyping in both groups.

It was revealed that the difference in the distribution of three different rs4977574 genotypes (AA, AG, and GG) between the control and general case group was significant (*p* = 0.036). The separate comparison of control subjects with LAS patients showed no significant difference in the distribution of rs4977574 genotypes (*p* = 0.162). At the same time, the frequency of rs4977574 genotypes in ACS patients significantly differed from the control group (*p* = 0.035).

The results of *ANRIL* rs4977574 genotypic association with the development of atherosclerosis and cardiovascular complications are shown in Table 4.

A significant association between rs4977574 locus and the risk of atherosclerosis complications (analysis in the general group) was found under the dominant (OR_obs_ = 1.436, CI 95% = 1.009‐2.044; *p*_obs_ = 0.044) and recessive (OR_obs_ = 1.551, CI 95% = 1.058‐2.273; *p*_obs_ = 0.025) models of inheritance. After adjusting for sex, age, body mass index, smoking, and hypertension, the association between rs4977574 locus and the risk of atherosclerosis complications remained only under the recessive model (*p*_adj_ = 0.048). Thus, individuals with the GG genotype had a 1.501-fold higher risk of atherosclerosis and cardiovascular complications (CI 95% = 1.003‐2.246) compared with A-allele carriers.

The link between rs4977574 polymorphism and the risk of LAS development was absent in all models of inheritance both before and after adjustment for covariates (*p* > 0.05). Instead, a significant relation between rs4977574 locus and the ACS was found under recessive inheritance model (OR_obs_ = 1.719, CI 95% = 1.110‐2.660; *p*_obs_ = 0.015). The statistical significance of the obtained results was preserved even after adjusting for nongenetic risk factors (*p*_adj_ = 0.049). The risk of ACS in individuals with GG genotype was 1.648 times (CI 95% = 1.002‐2.711) higher than in individuals with AA and AG genotypes.

A possible link between different *ANRIL* rs4977574 genotypes and lipid profile parameters in the case group was also analyzed (Table 5).

The results of ANOVA test in the general group revealed the association of rs4977574 locus with the serum concentration of total cholesterol (*p* = 0.021) and LDL (*p* = 0.022). The Bonferroni post hoc test showed a significant difference between GG and AA genotypes (*p* = 0.019, for total cholesterol; *p* = 0.025, for LDL). There was no relation between rs4977574 site and lipid profile parameters separately in LAS and ACS patients (*p* > 0.05).

## 4. Discussion

Thus, the relation between *ANRIL* gene rs4977574 polymorphism and the development of common atherosclerosis cardiovascular complications in the Ukrainian population was tested. The results in the general group revealed the significant association of rs4977574-GG genotype with increased risk of atherosclerosis lesions. A separate analysis in subgroups demonstrated that the rs4977574-GG genotype is linked to an increased risk of ACS, but not of LAS.

Over the past decade, a number of studies to determine the involvement of rs4977574 polymorphism in the development of various atherosclerosis complications have been published. Shanker et al. revealed that the G-A-A-A-A haplotype formed from five *ANRIL* gene polymorphic sites (rs1333049, rs10757278, rs2383206, rs4977574, and rs10757274, respectively) is associated with a two-fold reduction of the CAD risk in the Indian population [17]. The association between *ANRIL* gene rs4977574 locus and the occurrence of myocardial infarction in the Turkish population was revealed by Sakalar et al. [21]. Instead, Temel et al. did not find the link between rs4977574 polymorphism and CAD development in the Turkish population [18]. The results of a prospective cohort study in the Swedish population showed that the G-allele of the rs4977574 SNP increased the risk of ischemic stroke and myocardial infarction by 16% [20].

Studies in the Chinese population performed by Wang et al. demonstrated a strong association of the rs4977574 polymorphism with an increased risk of myocardial infarction, which persisted after adjustment for nongenetic risk factors [19]. The results of a case-control study by Huang et al. also showed a strong link between SNP rs4977574 and CAD development in the Chinese population [16]. Moreover, the authors also conducted a meta-analysis of the already published studies [29]. Obtained results confirmed the association of the G-allele with an increased risk of CAD occurrence. In the last few years, the results of three independent meta-analyses performed by Chinese researchers have also been published [24–26]. The significant link between *ANRIL* gene rs4977574 polymorphism and the development of CAD and myocardial infarction was reported.

In addition, Wang et al. performed both their own case-control study and meta-analysis to verify the relationship between the rs4977574 locus and ischemic stroke onset [22]. In contrast to our results, both analyses showed that the G-allele of rs4977574 SNP is related to an increased risk of ischemic stroke.

The results of our study showed the association between rs4977574-GG genotype and elevated serum concentrations of total cholesterol and LDL in patients with cardiovascular complications of atherosclerosis. Similar data were obtained by Temel et al. [18]. It was shown that the level of total cholesterol in the blood serum of CAD patients with rs4977574-GG genotype was significantly higher than in the main A-allele carriers. In addition, Hindy et al. reported that G-allele of rs4977574 locus was associated with reduced HDL serum levels in Swedes and nonsmokers [20]. Instead, no effect of rs4977574 locus on lipid profile in patients with myocardial infarction was detected by Wang et al. [19].

We have shown that the frequency of the rs4977574-G allele in the control group was 0.438, while in the common case group: 0.516. According to the 1000 Genomes project, the average frequency of G-alleles in the global population is 0.395; in Europeans: 0.492; in the population of both Americas: 0.416; in Central Asia: 0.531; in South Asia: 0.484; and in the African populations: 0.141 [26]. More detailed data from the European countries have shown that the G-allele frequency in Sweden population is 0.448 [20] and in the Finnish population: 0.355 [23]. Thus, the frequency of the G-allele of rs4977574 polymorphism in the Ukrainian population corresponds to this indicator in Europe and South Asia, and mostly in line with the Sweden population.

It is known that the polymorphic locus rs4977574 is located in the 16^th^ intron of the *ANRIL* gene (103785^th^ position). The question of the effect of this SNP on the transcription functioning of lncRNA ANRIL and the development of atherosclerotic phenotype remains debatable. According to the main hypothesis, it is assumed that the genotype of the rs4977574 intron locus may affect the balance between the formation of linear and circular ANRIL isoforms in proatherogenic cells, in particular, in macrophages and smooth muscle cells [7]. It is proposed that the presence of the G-allele leads to enhanced formation of linear isoforms of ANRIL molecule along with reduced expression of the circular ANRIL transcripts. The linear isoforms of the ANRIL molecule activate the PRC1, causing repression of tumor suppressors (CDKN2A and CDKN2B). Eventually, this leads to inhibition of apoptosis and excessive proliferation of proatherogenic cells. Instead, the A-allele may contribute to the enhanced formation of the circle ANRIL isoforms. Such type of ANRIL transcripts inhibits the activity of the PeBoW complex required for rRNA maturation. This in turn leads to rRNA deficiency, nucleolar stress, and p53 protein activation, culminating in the inhibition of cell division and apoptosis activation.

There are several limitations in our case-control study. The number of people enrolled in our study was relatively small. Moreover, persons treated in only two specific hospitals of one city were included. Thus, the association with LAS development, as well as with some lipid profile parameters could be missed due to small statistical power and weak population diversity. In addition, the relation between rs4977574 genotype and ANRIL isoform expression was not tested. However, we are going to perform such experiments in the near future. At the same time, we hope that the results of the present study will become an important part of the future meta-analysis of the link between *ANRIL* gene rs4977574 polymorphism and the development of atherosclerosis cardiovascular complications in European populations.

## 5. Conclusions

This is the first case-control study to analyze the relationship between *ANRIL* genetic polymorphism and cardiovascular disease development in the Ukrainian population. The obtained results showed that rs4977574 polymorphism is associated with atherosclerosis and may affect lipid profile. It was found that the rs4977574-GG genotype is linked to the increased risk of atherosclerosis and cardiovascular complications, and in particular, to the increase of ACS risk. However, no association between rs4977574 locus and the LAS development was established.

## Figures and Tables

**Table 1:** Baseline characteristics of the cases and controls.

	Controls *n* = 234	Atherosclerosis *n* = 395	*p*
Age (years)	66.1 ± 14.5	61.4 ± 11.0	<0.001
Female (%)	77 (32.9)	135 (34.2)	0.744
Male (%)	157 (67.1)	260 (65.8)	
Body mass index (kg/m^2^)	27.4 ± 4.7	28.1 ± 4.1	0.063
Body mass index ≥25 kg/m^2^ (%)	164 (70.1)	312 (79.0)	0.012
Systolic blood pressure (mmHg)	139.3 ± 23.1	154.8 ± 27.8	<0.001
Diastolic blood pressure (mmHg)	83.4 ± 10.7	93.0 ± 13.7	<0.001
Fasting glucose (mmol/l)	5.3 ± 0.7	6.9 ± 2.2	<0.001
Arterial hypertension (%)	73 (31.6)	268 (67.8)	<0.001
Smokers (%)	61 (26.1)	148 (37.5)	0.003

Note: *n*: case number. *χ*^2^-test and *t*-test were used for data comparison.

**Table 2:** Lipid profile in patients with atherosclerosis.

	LAS *n* = 187	ACS *n* = 195	Total *n* = 382	*p*
Total cholesterol (mmol/l)	4.98 ± 1.46	6.39 ± 1.40	5.70 ± 1.59	<0.001
LDL cholesterol (mmol/l)	3.17 ± 1.39	4.59 ± 1.49	3.89 ± 1.61	<0.001
HDL cholesterol (mmol/l)	1.01 ± 0.29	1.05 ± 0.22	1.03 ± 0.26	0.113
Triglyceride (mmol/l)	1.67 ± 0.77	1.66 ± 0.78	1.66 ± 0.77	0.890

Note: LAS: large artery stroke; ACS: acute coronary syndrome; LDL: low-density lipoproteins; HDL: high-density lipoproteins; *n*: case number. *t*-test was used for data comparison (LAS vs ACS).

**Table 3:** The frequency of *ANRIL* rs4977574 genotypes in the study groups.

Group	*n*	Genotype			*p*
		АА (%)	АG (%)	GG (%)	
Atherosclerosis (common group)					
Control	234	78 (33.3)	107 (45.7)	49 (20.9)	0.036
Case	395	102 (25.8)	178 (45.1)	115 (29.1)	

Large artery stroke					
Control	234	78 (33.3)	107 (45.7)	49 (20.9)	0.162
Case	200	52 (26.0)	94 (47.0)	54 (27.0)	

Acute coronary syndrome					
Control	234	78 (33.3)	107 (45.7)	49 (20.9)	0.035
Case	195	50 (25.6)	84 (43.1)	61 (31.3)	

Note: *n*: number of subjects. *χ*^2^-test was used for data comparison.

**Table 4:** Analysis of *ANRIL* rs4977574 genotypic association with the risk of atherosclerosis complications.

Model	*p*_obs_	OR_obs_ (95% CI)	*p*_adj_	OR_adj_ (95% CI)
Atherosclerosis (common group)				
AG+GG vs AA	0.044	1.436 (1.009-2.044)	0.185	1.286 (0.887-1.866)
GG vs AA+AG	0.025	1.551 (1.058-2.273)	0.048	1.501 (1.003-2.246)
AG vs AA+GG	0.872	0.974 (0.704-1.347)	0.600	0.912 (0.645-1.288)

Large artery stroke				
AG+GG vs AA	0.097	1.423 (0.938-2.159)	0.258	1.283 (0.833-1.974)
GG vs AA+AG	0.140	1.396 (0.896-2.176)	0.123	1.435 (0.907-2.270)
AG vs AA+GG	0.791	1.053 (0.721-1.537)	0.771	0.943 (0.634-1.402)

Acute coronary syndrome				
AG+GG vs AA	0.084	1.450 (0.952-2.209)	0.214	1.351 (0.840-2.171)
GG vs AA+AG	0.015	1.719 (1.110-2.660)	0.049	1.648 (1.002-2.711)
AG vs AA+GG	0.582	0.898 (0.613-1.317)	0.554	0.876 (0.565-1.358)

Note: 95% CI: 95% confidence interval; *p*_obs_: observed *p* value (unadjusted for covariates); OR_obs_: observed odds ratio; *p*_adj_: *p* value adjusted for sex, age, body mass index, smoking habit, and arterial hypertension; OR_adj_: odds ratio after adjusting for covariates.

**Table 5:** Stratified analysis of the link between *ANRIL* rs4977574 genotypes and lipid profile in patients with atherosclerosis.

	Genotype			*p*
	AA	AG	GG	
Atherosclerosis (common group)				
	*n* = 99	*n* = 170	*n* = 113	
Total cholesterol (mmol/l)	5.41 ± 1.57	5.67 ± 1.51	6.01 ± 1.70	0.021
LDL cholesterol (mmol/l)	3.64 ± 1.62	3.82 ± 1.51	4.22 ± 1.71	0.022
HDL cholesterol (mmol/l)	1.06 ± 0.26	1.04 ± 0.25	0.99 ± 0.29	0.144
Triglyceride (mmol/l)	1.52 ± 0.79	1.72 ± 0.76	1.71 ± 0.78	0.094

Large artery stroke				
	n = 49	n = 86	n = 52	
Total cholesterol (mmol/l)	4.73 ± 1.35	4.89 ± 1.40	5.38 ± 1.61	0.061
LDL cholesterol (mmol/l)	2.94 ± 1.28	3.07 ± 1.33	3.55 ± 1.55	0.059
HDL cholesterol (mmol/l)	1.04 ± 0.27	1.02 ± 0.29	0.96 ± 0.33	0.362
Triglyceride (mmol/l)	1.55 ± 0.76	1.64 ± 0.76	1.83 ± 0.80	0.161

Acute coronary syndrome				
	*n* = 50	*n* = 84	*n* = 61	
Total cholesterol (mmol/l)	6.08 ± 1.49	6.46 ± 1.16	6.55 ± 1.59	0.178
LDL cholesterol (mmol/l)	4.33 ± 1.63	4.60 ± 1.28	4.78 ± 1.63	0.253
HDL cholesterol (mmol/l)	1.08 ± 0.25	1.06 ± 0.19	1.02 ± 0.24	0.334
Triglyceride (mmol/l)	1.49 ± 0.82	1.79 ± 0.76	1.61 ± 0.75	0.082

Note: LDL: low-density lipoprotein; HDL: high-density lipoprotein, *n*: number of subjects. *F*-test and the Bonferroni post hoc test were used for data comparison.

## Data Availability

The results from this study have not been published in archives, databases, or repositories.
